The article "Mitigation of salinity stress in barley genotypes with variable salt tolerance by application of zinc oxide nanoparticles" was retracted in 2024. Reasons: compromised peer review; unreliable results or conclusions.

# Mitigation of salinity stress in barley genotypes with variable salt tolerance by application of zinc oxide nanoparticles

**DOI:** 10.3389/fpls.2022.973782

**Published:** 2022-08-22

**Authors:** Basharat Ali, Muhammad Hamzah Saleem, Shafaqat Ali, Munazzam Shahid, Muhammad Sagir, Muhammad Bilal Tahir, Kamal Ahmad Qureshi, Mariusz Jaremko, Samy Selim, Afzal Hussain, Muhammad Rizwan, Wajid Ishaq, M. Zia-ur Rehman

**Affiliations:** ^1^Khwaja Fareed University of Engineering and Information Technology (KFUEIT), Rahim Yar Khan, Pakistan; ^2^Faculty of Agriculture, University of Agriculture, Faisalabad, Pakistan; ^3^Institute of Crop Science and Resource Conservation (INRES), University of Bonn, Bonn, Germany; ^4^College of Plant Science and Technology, Huazhong Agricultural University, Wuhan, China; ^5^Department of Environmental Sciences and Engineering, Government College University Faisalabad, Faisalabad, Pakistan; ^6^Department of Biological Science and Technology, China Medical University, Taichung City, Taiwan; ^7^Department of Environmental Sciences, University of Jhang, Jhang, Pakistan; ^8^Department of Pharmaceutics, Unaizah College of Pharmacy, Qassim University, Unaizah, Saudi Arabia; ^9^Smart-Health Initiative (SHI) and Red Sea Research Center (RSRC), Division of Biological and Environmental Sciences and Engineering (BESE), King Abdullah University of Science and Technology (KAUST), Thuwal, Saudi Arabia; ^10^Department of Clinical Laboratory Sciences, College of Applied Medical Sciences, Jouf University, Sakaka, Saudi Arabia; ^11^Department of Environmental Sciences, The University of Lahore, Lahore, Pakistan; ^12^Nuclear Institute for Agriculture and Biology, Faisalabad, Pakistan

**Keywords:** salt stress, antioxidant machinery, oxidative stress, nanoparticles, barley, plant growth

## Abstract

Salinity has become a major environmental concern of agricultural lands, impairing crop production. The current study aimed to examine the role of zinc oxide nanoparticles (ZnO NPs) in reducing the oxidative stress induced by salinity and the overall improvement in phytochemical properties in barley. A total of nine different barley genotypes were first subjected to salt (NaCl) stress in hydroponic conditions to determine the tolerance among the genotypes. The genotype Annora was found as most sensitive, and the most tolerant genotype was Awaran 02 under salinity stress. In another study, the most sensitive (Annora) and tolerant (Awaran 02) barley genotypes were grown in pots under salinity stress (100 mM). At the same time, half of the pots were provided with the soil application of ZnO NPs (100 mg kg^–1^), and the other half pots were foliar sprayed with ZnO NPs (100 mg L^–1^). Salinity stress reduced barley growth in both genotypes compared to control plants. However, greater reduction in barley growth was found in Annora (sensitive genotype) than in Awaran 02 (tolerant genotype). The exogenous application of ZnO NPs ameliorated salt stress and improved barley biomass, photosynthesis, and antioxidant enzyme activities by reducing oxidative damage caused by salt stress. However, this positive effect by ZnO NPs was observed more in Awaran 02 than in Annora genotype. Furthermore, the foliar application of ZnO NPs was more effective than the soil application of ZnO NPs. Findings of the present study revealed that exogenous application of ZnO NPs could be a promising approach to alleviate salt stress in barley genotypes with different levels of salinity tolerance.

The article "Mitigation of salinity stress in barley genotypes with variable salt tolerance by application of zinc oxide nanoparticles" was retracted in 2024. Reasons: compromised peer review; unreliable results or conclusions.

## Introduction

Soil salinization is a rapidly growing agricultural problem, with an estimated 800 Mha of arable land currently damaged by salinity (Nachshon, 2018; Hussain et al., 2022). Increasing crop tolerance to salinity is a global priority because food production will need to keep up with rising global population demands (Amna et al., 2021; Ma et al., 2022). The effect of salinity on plant growth occurs in two phases: the first phase is dominated by osmotic stress and the second by ion-specific stress with a subsequent generation of free radicals and reactive oxygen species (ROS) (Ali et al., 2022a; Wahab et al., 2022). In the first phase, the accumulation of compatible solutes in the cytosol regulates osmotic adjustment in plant cells and helps maintain pressure potential, which is essential for normal cell function and growth (Hameed et al., 2021; Johnson et al., 2022).

Plants respond differently to salinity stress depending on species, genotype, and adaptability (Derbali et al., 2021). This deference determines the ability of plants to tolerate salinity and is reflected in their growth and development. Glycophytes are salt-sensitive plants that cannot tolerate higher concentrations of salinity, such as *Zea mays*, *Oryza sativa*, and *Glycine max*. At the same time, halophytes can endure salinity through their physiological, biochemical, and molecular mechanisms (Elsheery et al., 2020). Plants can adjust osmotic stress by decreasing the osmotic potential by accumulating osmolytes (Xue et al., 2021). The uptake of inorganic ions and the synthesis of organic solutes under stress conditions help plants to activate the antioxidant defense mechanism and prevent the denaturing of enzymes (Ali et al., 2022b,c). Plants have developed different signaling mechanisms, which enable them to tolerate salt stress, such as producing ROS, despite their toxic effect as signaling molecules in plant cells (Qian et al., 2021). Under salinity stress, the production of mitogen-activated protein kinase (MAPK) can trigger plant response to salinity by activating antioxidant enzymes (Qiao et al., 2021). Plants can sense hyperosmotic and ionic Na^+^ components of stress in combination with the Ca^+2^ channel and respond to them through their metabolic process (Ahmad and Akhtar, 2019). In plants, the calcium-permeable non-selective cation channels (NSCCs) restricts the Na^+^ influx, triggers K^+^ efflux, and contributes to efficient storage of Na^+^ in the vacuole (Zhao et al., 2020). The ability of plants to maintain K^+^ levels and control the exclusion of Na^+^ from photosynthetic leaves was highly efficient in enhancing the ability to tolerate salt stress (Aranda et al., 2021). In glycophytes, salinity tolerance is due to the ability of plants to have high osmo-tolerance coupled with tissue tolerance and a high ability to retain K^+^ in the mesophyll (Sarraf et al., 2022).

The article "Mitigation of salinity stress in barley genotypes with variable salt tolerance by application of zinc oxide nanoparticles" was retracted in 2024. Reasons: compromised peer review; unreliable results or conclusions.

It is considered that nanoparticles (NPs) can be used as a nutrient source, especially micronutrients (Arshad et al., 2021; Hazarika et al., 2022; Sarraf et al., 2022). Thus, the use of nano-fertilizers for the controlled release of concerning nutrients for crops might be a potential strategy to solve such issues of soil contamination and low agronomic productivity (Raliya et al., 2017). Among NPs, zinc oxide nanoparticles (ZnO NPs) are considered among the most highly used NPs in several industrial products (Sarraf et al., 2022). ZnO NPs have been suggested as a Zn fertilizer at lower levels to supply Zn to plants (Milani et al., 2012). It has been observed that ZnO NPs (1∼20 ppm) increase the growth of mung beans and chickpea (Mahajan et al., 2011). ZnO NPs have been found to enhance cotton growth and reduce oxidative stress in plants (Venkatachalam et al., 2017).

Barley is the fourth most important cereal crop after wheat, corn, and rice, which is cultivated worldwide to fulfill the food needs of humans and animals (Adnan et al., 2022; Farag et al., 2022). Barley is a salt-tolerant crop and has developed different morphological and chemical adaptions to endure salt stress. It can expel Na^+^ ions into the vacuole and prevent the accumulation of Na^+^ in the cytoplasm (Kreszies et al., 2019). High salinity may adversely affect the growth and yield of the barely crop (Pour-Aboughadareh et al., 2021). Different cultivars of the same species may differ in their growth response and intensity of damage under salt stress. This study was conducted to analyze the ability of nine different varieties of barley to endure salt stress and the ability of the nanoparticle to mitigate salt stress in barley plants. Furthermore, this study hypothesized that ZnO NPs may alleviate salinity stress in barley by enhancing Zn uptake and ultimately improving the morphological, physiological, and biochemical parameters. Overall, this study has provided new insights into the application of ZnO NPs for Zn bio-fortification and the effective role of ZnO NPs in mitigating the salinity stress in barley.

The article "Mitigation of salinity stress in barley genotypes with variable salt tolerance by application of zinc oxide nanoparticles" was retracted in 2024. Reasons: compromised peer review; unreliable results or conclusions.

## Materials and methods

### Plant material and growth conditions

A pot experiment was conducted in a wire house at the Institute of Soil and Environmental Sciences, University of Agriculture, Faisalabad, at 31° 25′ 59.55″ N, 73° 04′ 20″ E, 184.4 m above sea level. Following genotypes of barley from Pakistan and Germany were selected: V1 (Awaran 02), V2 (PK 30046), V3 (Sohrab 06), V4 (PK 30118), V5 (Acarda), V6 (PK 3019), V7 (Haider 95), V8 (Apex), and V9 (Annora). The seeds were germinated into moist quartz sand in a controlled chamber with a photoperiod of 16-h light/8-h dark and a light intensity of 225 ± 25 μmol m^–2^ s^–1^. The light/dark temperatures were set at 22°C/18°C, and relative humidity was set at 85%. For the experiment, 10-day-old six uniform seedlings were transferred to pots containing 5 L of water; each pot’s diameter was 35 cm and height 60 cm. For the first 4 days, the half-strength nutrient solution was given. After that, full strength nutrient solution was applied for the next 4 days. The nutrient solution was renewed every 4 days, and pots were continuously aerated with pumps. The applied nutrient solution contained MgSO_4_ (65.9 mg L^–1^), KNO_3_ (18.5 mg L^–1^), KH_2_PO_4_ (24.8 mg L^–1^), MnCl_2_. 4H_2_O (0.9 mg L^–1^), CuSO_4_. 5H_2_O (0.04 mg L^–1^), H_2_MoO_4_ (0.01 mg L^–1^), (NH_4_)_2_SO_4_ (48.2 mg L^–1^), K_2_SO_4_ (15.9 mg L^–1^), Ca (NO_3_)_2_ (59.9 mg L^–1^), Fe citrate (6.8 mg L^–1^), ZnSO_4_. 7H_2_O (0.11 mg L^–1^), and H_3_BO_3_ (2.9 mg L^–1^) (Sallah-Ud-Din et al., 2017). Different NaCl levels (50 and 100 mM) were maintained in corresponding pots by dissolving the required amount of salt to provide salinity stress to plants, as suggested by many researchers in their studies (Shams et al., 2019; Hawrylak-Nowak et al., 2021). Each treatment was replicated three times, and the experiment was designed according to a randomized complete block design. The pH of the solution was maintained at 6.5 every other day with 1 mol L^–1^ HCl or NaOH, as required.

In the first experiment, genotypes Awaran 02 and Annora were found as tolerant and sensitive, respectively, based on plant morphology, gas exchange attributes, and biochemical analysis. In the second experiment, these selected cultivars were used to assess the alleviating role of ZnO NPs on barley under salinity stress conditions. ZnO NPs were purchased from Alfa Aesar with a purity of 99%, 20–30 nm APS powder, and a density of 5.606. Surface sterilization of the selected barley cultivar seeds was carried out with sodium hypochlorite for 5 min and then washed thoroughly with distilled water. The experiment was conducted in a wire house at the Institute of Soil and Environmental Sciences, University of Agriculture, Faisalabad. A total of eight healthy and uniform-sized barley seeds (cvs. Annora and Awaran 02) were transferred to each plastic pot with 5.0 kg sand. The NaCl level (100 mM) was maintained in corresponding pots. For ZnO NPs exposure, half of the pots were treated with 100 mg kg^–1^ of ZnO NPs by thoroughly mixing, and barley seeds were sown after 15 days of ZnO NP application in the soil to avoid the immediate effects of NPs on seed germination. The remaining half pots were foliar sprayed with ZnO NPs (100 mg L^–1^) at different time intervals using Tween-20 as a sticking agent. Different treatments of ZnO NPs were prepared in distilled water and were ultrasonicated for about 30 min to separate and homogenize the particles. The growth conditions were kept the same as in the first experiment, and the pots were protected from rain during the entire growth period. The plants were thinned to five seedlings in each pot after 15 days of sowing, and the first foliar spray was carried out just after thinning the plants between 10 and 11 a.m., whereas second, third, and fourth foliar sprays were carried out at the fourth, sixth, and eighth weeks of sowing. During foliar spray, the soil of each pot and neighbor plants were covered to avoid direct entry of NPs to soil and surrounding plants due to foliar spray, whereas controlled plants were sprayed with distilled water simultaneously. A total volume of 2 L per treatment was used. In total, three replicates of each treatment were maintained in the experiment.

The article "Mitigation of salinity stress in barley genotypes with variable salt tolerance by application of zinc oxide nanoparticles" was retracted in 2024. Reasons: compromised peer review; unreliable results or conclusions.

### Plant harvesting and sampling

Barley plants were harvested at the vegetative stage. A stainless steel meter scale measured the plant height and root length. The plants were separated into leaves, shoots, and roots. The roots were washed with 0.1 M HCl to remove the ions on the root surface, and then, all the roots were carefully washed with distilled water. Oven drying of the samples was performed at 70°C for 72 h. The samples were crushed into small pieces after recording the dry weight and stored for ion analysis. Plant parameters including plant growth (plant height, root length, number of leaves per plant, and leaf area), plant biomass (dry weight of root and shoot), gas exchange attributes (transpiration rate, net photosynthetic rate, water use efficiency (WUE), and stomatal conductance), chlorophyll content (chlorophyll *a*, chlorophyll *b*, total chlorophyll, total carotenoids, and SPAD value), and accumulation of sodium ions in the root and shoot were measured according to standard protocols given as follows:

### Plant growth parameters

After 2 weeks of the treatment imposition, barley seedlings were harvested and carefully washed first with tap water and then with distilled water. Growth attributes like plant length, root length, number of leaves, root length, and leaf area were measured. The leaf area was measured by multiplying the length and width of the leaf. Plant parts, such as, root and shoot, were separated. Then, the plant samples were oven dried for 72 h at 70°C, and dry weights were recorded.

### Photosynthetic pigment contents

After 3 weeks of treatment, uppermost fully extended leaves were used to determine chlorophyll (Chl) and carotenoid contents. The pigment was extracted in 85% (v/v) acetone and kept under 4°C in darkness until leaf color disappeared and then centrifuged at 4,000 × *g* for a time duration of 10 min. The absorbance of the supernatant was recorded at 663, 644, and 452.5 nm for *Chl a*, *Chl b*, and carotenoids by using a spectrophotometer (JASCO V-730 UV-Visible) (Metzner et al., 1965). Chlorophyll and carotenoid contents were calculated by adjusting extinction coefficients and equations (Lichtenthaler and Buschmann, 2001). Finally, the contents of the pigments were given as mg g^–1^ fresh weights (FW).

### Gas exchange parameters

Gas exchange parameters, such as, stomatal conductance (gs), transpiration rate (E), photosynthetic rate (Pn), and WUE, were measured by using the infrared gas analyzer (IRGA) (LI-6200, Li-Cor Inc., Lincoln, NE, United States). The readings were taken on the topmost intact and fully expanded leaf after 2 h of acclimatization in a growth cabinet, at a temperature of 18°C, a light intensity of 1,000 μmol m^–2^ s^–1^, and relative humidity of 60%; at least eight readings per treatment were recorded (Ali et al., 2013).

### Ion analysis

Dry barley roots and shoots were ground and passed through a 2-mm mesh sieve. A 0.3 g weighed sample was digested in 10 mL 98% H_2_SO_4_ and 3 mL 30% H_2_O_2_ for 5 h, and the Na^+^ content was determined according to Skoog et al. (2000) by using a flame photometer (AA6300, Shimadzu, Tokyo, Japan).

### Analysis of lipid peroxidation and reactive oxygen species

The level of lipid peroxidation was measured in terms of the malondialdehyde (MDA) content determined by 2-thiobarbituric acid (TBA) reactive metabolites (Zhou and Leul, 1999). Fresh leaves and roots (0.2 g) were separately homogenized and extracted in 10 mL of 0.25% TBA made by 10% trichloroacetic acid (TCA). The extract was heated in water at 95°C for 30 min and then cooled on ice until room temperature. After centrifuging the extract at 5000 × *g* for 10 min, the absorbance of the supernatant was measured at 532 nm. Correction of non-specific turbidity was made by subtracting the absorbance value taken at 600 nm. The level of MDA was measured as μmol g^–1^ FW using an extinction coefficient of 155 mM cm^–1^.

The article "Mitigation of salinity stress in barley genotypes with variable salt tolerance by application of zinc oxide nanoparticles" was retracted in 2024. Reasons: compromised peer review; unreliable results or conclusions.

For determination of the hydrogen peroxide (H_2_O_2_) content, the samples (0.4 g) were extracted with 5.0 mL of TCA (0.1%, w/v) in an ice bath, and the homogenate was centrifuged at 12,000 × *g* for 15 min (Velikova et al., 2000). In 0.5 mL of the supernatant, 0.5 mL of phosphate buffer (pH 7.0) and 1.0 mL of potassium iodide (1 M) were added. The absorbance of the mixture was measured at 390 nm. The hydrogen peroxide content was determined using the extinction coefficient of 0.28 μM cm^–1^ and expressed as μmol g^–1^ DW.

### Determination of leaf and root electrolyte leakage

To determine the electrolyte leakage (EL), 100 g of fresh leaf samples were cut into 5-mm pieces and placed in test tubes containing deionized water. The leaf and root samples were incubated for 2 h at 32°C. After incubation, the tubes were cooled down, and EC_1_ was measured using the EC meter. After that, the solution was incubated again at 121°C for 20 min, and the procedure was revised for measuring EC_2_ (Mehmood et al., 2021). The EL was calculated using the following formula:


$$\text{EL}=\left({\text{EC}}_{1}/{\text{EC}}_{2}\right)\times 100$$

### Antioxidant enzymatic analysis

For biochemical analysis, the samples of roots and leaves (0.6 g) were homogenized in 8 mL of 50 mM potassium phosphate buffer (pH 7.8) under ice-cold conditions. The homogenate was centrifuged at 10,000 × *g* for 20 min at 4°C, and the supernatant was used to determine the following enzyme activities. The assay for ascorbate peroxidase (APX) (EC 1.11.1.11) activity was measured in a reaction mixture of 3 mL containing 100 mM phosphate (pH 7), 0.1 mM EDTA-Na_2_, 0.3 mM ascorbic acid, 0.06 mM H_2_O_2_, and 100 μL enzyme extract. The change in absorption was taken at 290 nm 30 s after adding H_2_O_2_ (Nakano and Asada, 1981). Catalase (CAT) (EC 1.11.1.6) activity was measured with the use of H_2_O_2_ (extinction coefficient 39.4 mM cm^–1^) for 1 min at A240 in 3 mL reaction mixture containing 50 mM potassium phosphate buffer (pH 7.0), 2 mM EDTA-Na_2_, 10 mM H_2_O_2_, and 100 μL enzyme extract (Zainab et al., 2021). Glutathione reductase (GR) (EC 1.6.4.2) activity was assayed by Jiang and Zhang (2001) with an oxidation of NADPH at 340 nm (extinction coefficient 6.2 mM cm^–1^) for 1 min. The reaction mixture comprised 50 mM potassium phosphate buffer (pH 7.0), 2 mM EDTA-Na_2_, 0.15 mM NADPH, 0.5 mM GSSG, and 100 μL enzyme extract in a volume of 1 mL. The reaction was started by using NADPH. Superoxide dismutase (SOD) (EC 1.15.1.1) activity was determined following the inhibition of photochemical reduction due to nitro blue tetrazolium (NBT) (Zhang et al., 2008). The reaction mixture comprised 50 mM potassium phosphate buffer (pH 7.8), 13 mM methionine, 75 μM NBT, 2 μM riboflavin, 0.1 mM EDTA, and 100 μL of enzyme extract in volume of 3 mL; one unit of SOD activity was measured as the amount of enzyme required to cause 50% inhibition of the NBT reduction measured at 560 nm. Peroxidase (POD) (EC1.11.1.7) activity was assayed by Zhou and Leul (1999) with some modifications. The reactant mixture contained 50 mM potassium phosphate buffer (pH 7.0), 1% guaiacol, 0.4% H_2_O_2_, and 100 μL enzyme extract. Variation due to guaiacol in absorbance was measured at 470 nm.

The article "Mitigation of salinity stress in barley genotypes with variable salt tolerance by application of zinc oxide nanoparticles" was retracted in 2024. Reasons: compromised peer review; unreliable results or conclusions.

### Statistical analysis

The replicated data from the experimental work were statistically analyzed by two-way analysis of variance (ANOVA) through SPSS^®^ Statistics version 25 to determine the significant variance. The means were compared through the *post-hoc* test, followed by the Tukey test. The *p*-value was perceived to be significant at ≤0.05.

## Results

### Effects of NaCl stress on barley seedlings

#### Effects on plant morphology

The obtained values of plant growth traits (shoot and root length, number of leaves, leaf area, and shoot and root dry weight) notably declined with the increasing NaCl concentration (Supplementary Table 1). A significant reduction and severe toxic effects were revealed at an excessive NaCl level (100 mM) compared to 50 mM and control treatments in all nine genotypes. Maximum reduction in plant growth parameters was noted in the Annora genotype, and minimum reduction was noticed in the Awaran 02 genotype. Overall, the results revealed that Annora was the most sensitive cultivar, and Awaran 02 genotype was found to be the most tolerant genotype at all given concentrations of NaCl (Supplementary Table 1).

#### Effects on photosynthetic pigments

Chlorophyll (Chl) and carotenoid contents in the leaves of various barley genotypes were quantified in order to estimate the potential effects of NaCl on photosynthetic traits (Supplementary Table 2). The values of *Chl a*, *Chl b*, and carotenoid contents decreased significantly with increasing NaCl levels. The maximum reduction in Chl and carotenoids attributes was noted under the highest dose of NaCl (100 mM). Among all genotypes, the Annora genotype showed maximum reduction in Chl and carotenoid levels, while minimum reduction among these parameters was noticed in the Awaran 02 genotype (Supplementary Table 2).

The article "Mitigation of salinity stress in barley genotypes with variable salt tolerance by application of zinc oxide nanoparticles" was retracted in 2024. Reasons: compromised peer review; unreliable results or conclusions.

#### Effects on gas exchange parameters

To get insights into the physiological alteration, the leaf gas exchange parameters (photosynthetic rate, transpiration rate, stomatal conductance, and WUE) were analyzed under different NaCl concentrations (50 and 100 mM) in the nine barley genotypes (Table 1). All genotypes, except Annora, showed slight decreases in gas exchange traits at 50 mM NaCl compared to the control treatment. Under 100 mM NaCl, the maximum reduction in gas exchange parameters was found in the Annora genotype as compared to other treatments and genotypes. Among all studied genotypes, the Awaran 02 genotype experienced the least decline, and V9 showed the maximum decline in gas exchange parameters (Table 1).

**TABLE 1:** Effect of different concentrations of NaCl on gas exchange parameters of different barley genotypes.

Parameters	Na^+^ Level	Varieties								
		V1	V2	V3	V4	V5	V6	V7	V8	V9
Net photosynthesis rate (μmol CO_2_ m^–2^ s^–1^)	0	5.24^abc^ (0.20)	5.06^bcde^ (0.15)	4.95^efg^ (0.19)	5.25^abc^ (0.11)	5.01^defg^ (0.28)	5.34^ab^ (0.11)	5.20^ab^ (0.08)	5.42^abcd^ (0.16)	5.08^bcde^ (0.15)
	50	4.90^fg^ (0.14)	4.76^gh^ (0.10)	4.63^h^ (0.09)	4.28^i^ (0.23)	4.06^ik^ (0.24)	3.93^jk^ (0.15)	3.72^kl^ (0.15)	3.59^lm^ (0.09)	3.27^no^ (0.20)
	100	3.71^kl^ (0.10)	3.54^lm^ (0.07)	3.42^mn^ (0.13)	3.28^no^ (0.13)	3.10^op^ (0.12)	2.99^p^ (0.08)	2.73^q^ (0.17)	2.61^q^ (0.07)	2.48^q^ (0.10)
Transpiration rate (mmol H_2_O m^–2^ s^–1^)	0	2.56^ab^ (0.09)	2.48^bc^ (0.07)	2.56^ab^ (0.10)	2.47^bc^ (0.07)	2.60^ab^ (0.05)	2.54^cd^ (0.04)	2.39^ab^ (0.08)	2.57^ab^ (0.04)	2.41^cd^ (0.09)
	50	2.38^cd^ (0.07)	2.30^de^ (0.07)	2.20^e^ (0.06)	2.06^f^ (0.12)	1.93^g^ (0.07)	1.74^hi^ (0.05)	1.67^i^ (0.06)	1.53^jk^ (0.06)	1.45^kl^ (0.06)
	100	1.93^g^ (0.08)	1.84^gh^ (0.04)	1.73^hi^ (0.05)	1.64^ij^ (0.04)	1.55^jk^ (0.04)	1.48^kl^ (0.02)	1.38^lm^ (0.05)	1.32^mn^ (0.02)	1.25^n^ (0.02)
Stomatal conductance (mol m^–2^ s^–1^)	0	2.27^a^ (0.05)	2.21^ab^ (0.03)	2.10^cd^ (0.08)	2.23^ab^ (0.05)	2.15^bc^ (0.06)	2.13^bcd^ (0.12)	2.31^a^ (0.07)	2.23^ab^ (0.09)	2.16^bc^ (0.06)
	50	2.14^bcd^ (0.04)	2.09^cd^ (0.03)	2.04^d^ (0.06)	1.92^e^ (0.06)	1.88^ef^ (0.07)	1.80^f^ (0.07)	1.65^g^ (0.05)	1.60^gh^ (0.03)	1.51^hij^ (0.06)
	100	1.59^gh^ (0.09)	1.54^hi^ (0.04)	1.47^ijk^ (0.06)	1.42^jk^ (0.04)	1.37^kl^ (0.04)	1.32^lm^ (0.03)	1.22^mn^ (0.05)	1.16^no^ (0.03)	1.09^o^ (0.06)
Water use efficiency (%)	0	8.87^bcd^ (0.26)	8.78^bcd^ (0.49)	9.50^a^ (0.28)	9.18^ab^ (0.35)	8.90^bcd^ (0.26)	9.35^a^ (0.19)	9.12^abc^ (0.14)	8.67^cd^ (0.33)	9.19^ab^ (0.200)
	50	8.88^bcd^ (0.39)	8.48^d^ (0.19)	8.00^e^ (0.22)	7.57^f^ (0.17)	7.15^g^ (0.18)	6.84^gh^ (0.11)	6.38^ij^ (0.24)	6.09^jk^ (0.11)	5.75^klm^ (0.26)
	100	6.64^hi^ (0.19)	6.45^hij^ (0.14)	6.28^ij^ (0.12)	5.80^kl^ (0.31)	5.50^lm^ (0.33)	5.32^mn^ (0.21)	5.04^no^ (0.20)	4.86^o^ (0.12)	4.43^p^ (0.28)

Values are expressed as means of three replicates with standard deviations.

The article "Mitigation of salinity stress in barley genotypes with variable salt tolerance by application of zinc oxide nanoparticles" was retracted in 2024. Reasons: compromised peer review; unreliable results or conclusions.

Different letters indicate that values are significantly different at *p* < 0.05.

#### Effects on oxidative stress

Under non-stress conditions, no significant differences in the contents of malondialdehyde (MDA), hydrogen peroxide (H_2_O_2_), and leaf and root EL were observed in different barley genotypes (Table 2). The highest increase in the MDA and H_2_O_2_ contents was noted in the roots and leaves of all genotypes at 100 mM NaCl as compared to the control. The contents of MDA and H_2_O_2_ were higher in the V9 genotype than in other genotypes (Table 2). All genotypes showed maximum increases in EL at 100 mM NaCl as compared to 50 mM NaCl and control. The maximum and minimum EL levels were noticed in V9 and V1 genotypes under 100 mM NaCl and control treatments, respectively (Table 2).

**TABLE 2:** Effect of different concentrations of NaCl on oxidative stress of different barley genotypes.

Parameter	Na^+^ Level	Varieties								
		V1	V2	V3	V4	V5	V6	V7	V8	V9
MDA in leaves (μmol g^–1^ FW)	0	17.51^kl^ (0.26)	16.48^l^ (0.52)	16.65^l^ (0.64)	18.25^jk^ (0.54)	17.09^kl^ (0.49)	17.76^jkl^ (0.27)	17.64*^kl^* (0.67)	17.03^kl^ (0.49)	17.96^jkl^ (0.37)
	50	18.16^jk^ (1.22)	19.16^ij^ (0.55)	19.64^hi^ (0.71)	21.88^fg^ (0.55)	22.68^ef^ (0.91)	23.67^e^ (0.91)	25.31^d^ (0.95)	25.57^d^ (0.74)	26.51^cd^ (0.58)
	100	20.69^gh^ (0.52)	21.43^fg^ (0.86)	22.62^ef^ (0.90)	23.61^e^ (0.91)	25.25^d^ (0.95)	26.97^c^ (1.55)	28.82^b^ (0.75)	29.99^ab^ (0.86)	31.05^a^ (1.19)
MDA in roots (μmol g^–1^ FW)	0	23.25^lm^^(^0.51)	22.43^lm^ (0.65)	22.21^m^ (1.25)	24.03^klm^ (0.71)	23.22^lm^ (0.89)	22.50^lm^ (0.65)	23.65^lm^ (0.49)	23.05^lm^ (0.35)	21.93^m^ (0.84)
	50	23.37^lm^ (0.98)	24.59^kl^ (0.64)	25.73^k^ (1.60)	28.21^j^ (0.71)	29.22^ij^ (1.17)	30.90^hi^ (1.22)	32.23^fgh^ (1.26)	33.38^ef^ (0.65)	34.97^e^ (0.99)
	100	29.82^ij^ (1.14)	31.07^fhi^ (1.55)	33.01^efg^ (0.86)	34.54^e^ (2.15)	38.10^d^ (0.74)	40.16^c^ (1.01)	41.61^bc^ (1.66)	43.43^b^ (1.67)	45.87^a^ (1.76)
H_2_O_2_ in leaves (μmol g^–1^ FW)	0	5.70^klm^ (0.12)	5.56^lm^ (0.08)	5.24^m^ (0.16)	5.29^m^ (0.20)	5.80^kl^ (0.17)	5.43^lm^ (0.16)	5.64^klm^ (0.09)	5.60^lm^ (0.21)	5.41^lm^ (0.16)
	50	5.87^kl^ (0.15)	6.08^jk^ (0.24)	6.42^ij^ (0.26)	6.70^i^ (0.26)	7.17^h^ (0.27)	7.66^g^ (0.44)	8.18^ef^ (0.21)	8.51^de^ (0.25)	8.81^d^ (0.34)
	100	7.45^gh^ (0.19)	7.80^fg^ (0.41)	8.16^ef^ (0.32)	8.89^d^ (0.47)	9.55^c^ (0.25)	9.87^c^ (0.19)	10.34^b^ (0.29)	10.71^ab^ (0.27)	10.87^a^ (0.24)
H_2_O_2_ in root (μmol g^– 1^ FW)	0	8.39^kl^ (0.32)	8.10^kl^ (0.23)	7.92^l^ (0.30)	8.39^kl^ (0.18)	8.02^l^ (0.45)	8.54^kl^ (0.18)	8.32^kl^ (0.13)	8.68^jkl^ (0.26)	8.12^kl^ (0.23)
	50	8.87^jk^ (0.55)	9.72^i^ (0.25)	10.07^hi^ (0.40)	10.65^gh^ (0.42)	11.01^fg^ (0.65)	11.60^ef^ (0.62)	12.56^d^ (0.24)	12.90^d^ (0.28)	13.29^d^ (0.38)
	100	9.36^ij^ (0.46)	9.89^i^ (0.42)	10.78^gh^ (0.38)	11.82^e^ (0.71)	13.31^d^ (0.77)	14.22^c^ (0.37)	14.83^bc^ (0.47)	15.37^ab^ (0.44)	15.89^a^ (0.53)
EL in leaves (%)	0	25.68^no^ (0.76)	24.05^nopq^ (0.69)	24.99^nopq^ (0.38)	24.82^nopq^ (0.95)	23.97^opq^ (0.69)	25.27^nop^ (0.53)	24.63^nopq^ (0.37)	23.20^q^ (0.73)	23.43^pq^ (0.90)
	50	26.02^n^ (1.62)	28.53^m^ (0.72)	29.56^klm^ (1.18)	31.25^jk^ (1.23)	32.31^ij^ (1.91)	34.05^hi^ (1.82)	36.85^ef^ (0.71)	37.86^def^ (0.83)	39.00^cd^ (1.120)
	100	29.04^lm^ (1.33)	30.77^jkl^ (0.55)	32.22^ij^ (1.24)	34.53^gh^ (0.56)	36.11^fg^ (0.91)	38.23^de^ (0.84)	40.38^c^ (1.12)	42.85^b^ (0.96)	44.86^a^ (1.96)
EL in root (%)	0	35.90^klm^ (1.37)	34.68^lm^ (1.00)	33.90^m^ (1.30)	35.94^klm^ (0.79)	34.33^lm^ (1.93)	36.56^klm^ (0.76)	35.64^lm^ (0.54)	37.15^kl^ (1.10)	34.78^lm^ (1.00)
	50	38.66^jk^ (1.14)	40.61^j^ (1.17)	44.46^i^ (1.78)	46.40h^i^ (1.78)	47.46^h^ (1.37)	51.43^g^ (1.00)	54.22^f^ (1.37)	56.17^ef^ (2.24)	58.33^e^ (2.25)
	100	54.09^f^ (2.09)	57.07^e^ (1.25)	58.79^e^ (1.69)	64.35^d^ (2.57)	67.16^c^ (2.58)	68.71^c^ (1.98)	72.81^b^ (2.10)	74.59^ab^ (1.13)	76.52^s^ (1.59)

Values are expressed as means of three replicates with standard deviations.

The article "Mitigation of salinity stress in barley genotypes with variable salt tolerance by application of zinc oxide nanoparticles" was retracted in 2024. Reasons: compromised peer review; unreliable results or conclusions.

Different letters indicate that values are significantly different at *p* < 0.05.

#### Effects on antioxidant machinery

Data regarding the activities of ROS-detoxifying antioxidant enzymes such as SOD, peroxidase dismutase (POD), CAT, and APX in the leaves and roots of the nine genotypes under different concentrations of NaCl are given in Table 3. Significant alterations were observed in the activities of antioxidant enzymes in plant tissues of barley genotypes under different NaCl treatments compared to control treatments. At 100 mM NaCl, SOD activity in the root and leaf tissues decreased significantly in all genotypes of barley as compared to their respective control. The maximum decline in SOD activity was observed in leaves and roots of the V9 genotype under 100 mM NaCl treatments. Similarly, POD activity displayed decreasing trends with the increasing concentration of salinity. Compared to controls, POD activity significantly declined under 100 mM NaCl treatments in all genotypes, except for V1 and V2 genotypes, in which POD activity did not illustrate any significant difference in values (Table 3). A gradual decline in CAT activity was observed with an increasing concentration of salinity in all genotypes of barley. Minimum CAT activities were recorded in the leaves and roots of all nine genotypes at 100 mM of NaCl. The APX activity linearly declined in the shoots and roots of all genotypes with an increasing concentration of salinity. The minimum APX activity was found in both the leaves and roots of the V9 genotype under 100 mM NaCl concentration compared to other genotypes (Table 3).

The article "Mitigation of salinity stress in barley genotypes with variable salt tolerance by application of zinc oxide nanoparticles" was retracted in 2024. Reasons: compromised peer review; unreliable results or conclusions.

**TABLE 3:** Effect of different concentrations of NaCl on the contents of antioxidant enzyme activities of different barley genotypes.

Parameters	Na^+^ Level	Varieties								
		V1	V2	V3	V4	V5	V6	V7	V8	V9
SOD in leaves (Units g^–1^ FW)	0	132.73^ab^ (2.01)	124.98^cd^ (3.92)	134.64^ab^ (2.04)	126.25^cd^ (4.84)	133.90^ab^ (4.50)	129.56^bc^ (3.73)	133.71^ab^ (5.11)	129.15^bc^ (3.72)	136.16^a^ (2.83)
	50	128.77^bc^ (4.94)	121.90^de^ (4.67)	116.80^ef^ (4.67)	112.73*^f^* (2.84)	106.94^g^ (2.07)	96.96^h^ (6.03)	92.67^hij^ (2.40)	87.22^jkl^ (4.35)	83.72^klm^ (3.21)
	100	94.24^h^ (1.96)	91.87^hij^ (1.39)	89.67^ijk^ (2.58)	84.62^klm^ (2.44)	82.72^lm^ (3.17)	79.26^m^ (3.17)	72.41^n^ (2.09)	70.29^n^ (1.53)	66.62^n^ (2.57)
SOD in roots (Units g^–1^ FW)	0	178.92^ab^ (6.84)	173.37^bc^ (4.99)	182.20^a^ (3.79)	177.61^abc^ (2.68)	168.94^cd^ (6.84)	179.12^ab^ (3.92)	172.82^bc^ (4.98)	171.11^bcd^ (9.61)	185.16^a^ (5.48)
	50	171.69^bcd^ (7.49)	163.97^d^ (3.68)	154.51^e^ (4.30)	146.29^f^ (3.22)	138.20^g^ (3.49)	132.15^gh^ (2.12)	123.29^ij^ (4.73)	117.76^jk^ (2.12)	111.12^kl^ (5.07)
	100	133.21^gh^ (3.89)	128.50^hi^ (4.04)	123.18^ij^ (3.21)	115.30^jkl^ (6.63)	107.96^l^ (4.04)	97.39^m^ (2.81)	93.44^mn^ (3.26)	85.70^no^ (3.62)	81.11^o^ (3.98)
POD in leaves (Units g^–1^ FW)	0	314.32^cdef^ (9.06)	311.20^cdef^ (17.49)	336.76^a^ (9.97)	325.41^abcd^ (12.43)	315.31^bcdef^ (9.08)	331.37^ab^ (6.89)	323.03^abcde^ (4.88)	3.7.25^ef^ (11.78)	325.77^abc^ (7.13)
	50	316.68^bcdef^ (6.59)	308.71^def^ (4.66)	301.33^f^ (8.68)	284.36^g^ (8.20)	277.97^gh^ (10.66)	266.34^hi^ (10.64)	243.31^jk^ (7.01)	236.18^jklm^ (5.15)	223.88^lmn^ (8.64)
	100	252.05^ij^ (9.66)	238.61^jkl^ (9.15)	228.63^klm^ (9.14)	220.66^mn^ (5.56)	209.32^n^ (4.06)	189.79^o^ (11.81)	181.38^op^ (4.70)	170.72^pq^ (8.51)	163.87^q^ (6.28)
POD in root (Units g^– 1^ FW)	0	457.04^abc^ (17.46)	441.45^bcde^ (12.73)	431.53^def^ (16.55)	457.54^abc^ (10.02)	437.08^cdef^ (24.56)	465.40^ab^ (9.68)	453.69^abcd^ (6.86)	472.98^a^ (14.00)	442.84^bcde^ (12.76)
	50	439.92^cdef^ (12.67)	427.03^ef^ (9.32)	415.70^f^ (8.06)	384.11^g^ (20.50)	364.11^gh^ (21.55)	352.50^hi^ (13.89)	333.40^ij^ (13.32)	321.78^jk^ (8.11)	293.54^lm^ (18.26)
	100	325.27^j^ (9.17)	310.53^jkl^ (6.05)	299.80^kl^ (11.70)	287.41^lm^ (11.33)	271.84^mn^ (11.33)	262.36^n^ (6.62)	239.34^o^ (14.89)	228.74^o^ (5.93)	217.38^o^ (9.13)
CAT in leaves (Units g^– 1^ FW)	0	81.71^ab^ (1.70)	79.65^abcd^ (1.20)	75.00^e^ (2.36)	75.76^de^ (2.90)	83.04^a^ (2.46)	77.75^bcde^ (2.24)	80.80^ab^ (1.22)	80.24^abc^ (3.07)	77.50^bcde^ (2.23)
	50	76.50^cde^ (2.21)	75.72^de^ (2.84)	70.79^f^ (2.71)	67.83^fg^ (2.71)	64.26^ghi^ (2.57)	62.02^hij^ (1.56)	58.33^jkl^ (1.14)	55.62^lm^ (2.99)	51.32^no^ (3.23)
	100	65.86^gh^ (2.52)	63.61^hi^ (1.83)	61.12^ijk^ (1.59)	57.21^klm^ (3.29)	53.56^mn^ (2.01)	50.08^no^ (1.92)	47.98^op^ (1.92)	45.46^pq^ (1.82)	43.87^q^ (1.11)
CAT in root (Units g^– 1^ FW)	0	106.42^ab^ (4.07)	102.79^abcd^ (2.96)	101.77^bcd^ (5.72)	100.48^cd^ (3.85)	106.54^ab^ (2.33)	108.37^a^ (2.25)	105.64^abc^ (1.60)	103.11^abcd^ (2.97)	107.83^a^ (2.18)
	50	102.95^abcd^ (3.95)	98.64^de^ (3.94)	95.20^e^ (2.40)	90.31^f^ (1.75)	83.35^g^ (2.40)	81.48^ghi^ (3.12)	78.07^hij^ (3.12)	71.32^kl^ (2.05)	67.89^lm^ (2.01)
	100	86.67^fg^ (1.90)	83.63^g^ (2.41)	82.77^gh^ (3.10)	77.39^ij^ (2.97)	74.15^jk^ (2.96)	71.15^kl^ (1.80)	64.22^mn^ (2.31)	62.65^n^ (1.81)	59.40^n^ (3.98)
APX in leaves (Units g^– 1^ FW)	0	444.74^bcde^ (12.81)	467.40^ab^ (9.27)	455.64^abcd^ (6.88)	433.38^def^ (16.62)	459.50^abc^ (10.06)	443.35^cde^ (12.78)	438.95^cde^ (24.67)	475.01a (14.06)	459.00^abc^ (17.45)
	50	438.37^cde^ (12.63)	425.52^ef^ (9.29)	414.23^f^ (8.03)	382.75^g^ (20.43)	363.13^gh^ (21.47)	351.25^hi^ (13.85)	332.22^ij^ (13.27)	320.64^jk^ (8.09)	292.50^lm^ (18.20)
	100	305.08^kl^ (13.31)	291.37^lm^ (6.54)	274.56^mn^ (7.64)	259.94^no^ (5.73)	245.94^op^ (6.20)	234.82^pq^ (3.78)	219.08^qr^ (8.40)	209.25^r^ (3.76)	197.44^r^ (9.20)
APX in root (Units g^–1^ FW)	0	643.96^abc^ (14.10)	621.32^cde^ (17.92)	615.16^cde^ (34.57)	665.69^a^ (19.71)	643.26^abc^ (24.58)	623.28^bcde^ (17.95)	655.03^ab^ (13.63)	638.55^abcd^ (9.65)	607.35^de^ (23.29)
	50	613.79^cde^ (33.96)	594.38^ef^ (16.48)	568.13^fg^ (21.71)	550.49^gh^ (15.86)	531.04^hi^ (16.68)	509.07^i^ (13.28)	472.97^j^ (18.13)	448.85^jkl^ (11.71)	420.14^lmn^ (24.17)
	100	459.18^jk^ (20.03)	438.55^klm^ (9.84)	413.24^mn^ (11.50)	391.25^no^ (8.62)	369.62^op^ (9.32)	353.43^pq^ (5.68)	329.75^qr^ (12.64)	314.94^rs^ (5.66)	297.18^s^ (13.57)

Values are expressed as means of three replicates with standard deviations.

The article "Mitigation of salinity stress in barley genotypes with variable salt tolerance by application of zinc oxide nanoparticles" was retracted in 2024. Reasons: compromised peer review; unreliable results or conclusions.

Different letters indicate that values are significantly different at *p* < 0.05.

#### Effects on endogenous Na^+^ contents

Sodium ion (Na^+^) contents in the roots and shoots increased linearly with NaCl concentration (Table 4). An increasing trend in Na^+^ contents was found in both leaves and roots. In leaves, maximum Na^+^ accumulation was noticed in the V9 genotype, followed by V8>V7>V6>V5>V4>V3>V2>V1 under 100 mM NaCl (Table 4). Similar increasing trends in Na^+^ levels were noticed in barley roots. The Annora genotype showed the maximum accumulation of the Na^+^ content under 100 mM NaCl. The results proved that the Annora genotype was more sensitive to NaCl stress than all other genotypes due to the maximum accumulation of Na^+^ in the genotype. The least Na^+^ accumulation was noticed in the Awaran 02 genotype, depicting it as the most tolerant genotype (Table 4).

**TABLE 4:** Effect of different concentrations of NaCl on uptake of Na^+^ of different barley genotypes.

Parameters	Na^+^ Level	Varieties								
		V1	V2	V3	V4	V5	V6	V7	V8	V9
Na^+^ in shoot (mg g^– 1^ DW)	0	30.34^n^ (0.63)	29.58^n^ (0.45)	30.84^n^ (0.91)	28.87^n^ (0.83)	29.80^n^ (1.14)	28.78^n^ (0.83)	28.13^n^ (1.08)	29.83^n^ (0.65)	28.49^n^ (1.60)
	50	102.53^m^ (4.09)	107.92^m^ (3.92)	114.75^l^ (3.12)	129.73^k^ (3.16)	141.58^ij^ (5.66)	147.76^hi^ (5.67)	160.18^g^ (4.61)	164.10^fg^ (2.48)	168.34^f^ (3.50)
	100	138.55^j^ (2.81)	143.43^ij^ (4.24)	150.67^h^ (4.34)	167.03^fg^ (4.52)	176.09^e^ (5.08)	190.80^d^ (3.70)	201.14^c^ (5.07)	208.40^b^ (8.33)	217.50^a^ (8.34)
Na^+^ in root (mg g^– 1^ DW)	0	12.18^m^ (0.18)	12.10^m^ (0.46)	11.69^m^ (0.34)	12.32^m^ (0.26)	12.01^m^ (0.18)	11.31^m^ (0.36)	11.42^m^ (0.44)	12.52^m^ (0.37)	11.72^m^ (0.34)
	50	49.17^l^ (1.65)	51.96^kl^ (3.23)	55.25^k^ (2.00)	62.39^j^ (2.46)	64.50^ij^ (3.81)	67.99^hi^ (3.63)	73.58^g^ (1.43)	75.59^fg^ (1.65)	77.87^f^ (2.24)
	100	67.32^i^ (3.28)	71.63^gh^ (3.11)	78.25^f^ (3.03)	88.35^e^ (2.90)	94.98^d^ (2.39)	102.71^c^ (3.94)	109.85^b^ (4.12)	110.99^b^ (3.20)	115.03^a^ (2.52)

Values are expressed as means of three replicates with standard deviations.

Different letters indicate that values are significantly different at *p* < 0.05.

### Stress tolerance in barley genotypes by zinc oxide nanoparticles

#### Effects of zinc nanoparticles on plant morphology

The results pertaining to shoot length, root length, number of leaves per plant, leaf area, shoot dry weight, and root dry weight are shown in Figure 1. In both genotypes, a significant reduction was found in shoot and root length under salinity stress. However, both shoot and root length significantly enhanced when ZnO NPs were applied in soil or foliar spray under salinity stress. Moreover, ZnO NPs application significantly increased the number of leaves and leaf area in both cultivars under salinity stress. Moreover, ZnO NP application also significantly improved dry biomass in both cultivars under salinity. At the foliar application of ZnO NPs (100 mg L^–1^), higher dry weights of shoots and roots were found than in soil application in both cultivars (Figure 1).

The article "Mitigation of salinity stress in barley genotypes with variable salt tolerance by application of zinc oxide nanoparticles" was retracted in 2024. Reasons: compromised peer review; unreliable results or conclusions.

**FIGURE 1:** Effects of different concentrations of NaCl (0 and 100 mM) and ZnO NPs (0, 100 mg kg^–1^ soil, and 100 mg L^–1^ foliar) on **(A)** shoot length, **(B)** root length, **(C)** number of leaves per plant, **(D)** leaf area, **(E)** shoot dry weight, and **(F)** root dry weight of two barley genotypes Annora (salt sensitive) and Awaran 02 (salt tolerant). Values are expressed as means of three replicates with standard deviations. Different letters indicate that values are significantly different at a *p*-value < 0.05.

#### Effects of zinc nanoparticles on photosynthetic pigments

Chlorophyll and carotenoid concentrations were significantly increased in both foliar and soil applications of ZnO NPs as compared to the respective control treatments (Figure 2). The increasing concentration of ZnO NPs increased the chlorophyll and carotenoid contents, despite the increasing concentration of salinity in both genotypes. The maximum increase in chlorophyll and carotenoid contents was noticed in the tolerant Awaran 02 genotype as compared to the sensitive Annora genotype with the foliar application of ZnO NPs at 100 mM salinity level (Figure 2).

**FIGURE 2:** Effects of different concentrations of NaCl (0 and 100 mM) and ZnO NPs (0, 100 mg kg^–1^ soil, and 100 mg L^–1^ foliar) on **(A)** chlorophyll a, **(B)** chlorophyll b, **(C)** total chlorophyll, **(D)** carotenoid contents, **(E)** Na^+^ uptake in shoots, and **(F)** Na^+^ uptake in roots of two barley genotypes Annora (salt sensitive) and Awaran 02 (salt tolerant). Values are expressed as means of three replicates with standard deviations. Different letters indicate that the values are significantly different at a *p*-value < 0.05.

#### Effects of zinc nanoparticles on endogenous Na^+^ contents

To investigate the effects of ZnO NPs on Na^+^ concentrations, uptake of Na^+^ in barley shoots and roots was determined (Figure 2). The highest Na^+^ concentrations were observed in the plants grown under 100 mM salinity stress. Among the cultivars, more Na^+^ concentration was found in the sensitive Annora genotype than in the tolerant Awaran 02 genotype. Foliar and soil application of ZnO NPs decreased Na^+^ uptake in shoots and roots, despite the increasing concentration of salinity. The maximum decrease in Na^+^ uptake was observed by the foliar application of ZnO NPs than the soil application of ZnO NPs in both genotypes (Figure 2).

#### Effects of zinc nanoparticles on gas exchange attributes

The photosynthetic rate and transpiration rate were significantly reduced under salinity stress in both cultivars, and a maximum decrease in the photosynthetic rate and transpiration rate was observed in the Annora cultivar (Figure 3). However, photosynthetic and transpiration rates were significantly enhanced when ZnO NPs were applied in soil or foliar spray under salinity stress. A maximum increase in gas exchange parameters was found with foliar application of ZnO NPs in the Awaran 02 genotype. Furthermore, ZnO NP application also significantly improved the stomatal conductance and WUE in both cultivars under salinity stress (Figure 3).

The article "Mitigation of salinity stress in barley genotypes with variable salt tolerance by application of zinc oxide nanoparticles" was retracted in 2024. Reasons: compromised peer review; unreliable results or conclusions.

**FIGURE 3:** Effects of different concentrations of NaCl (0 and 100 mM) and ZnO NPs (0, 100 mg kg^–1^ soil, and 100 mg L^–1^ foliar) on **(A)** net photosynthesis rate, **(B)** transpiration rate, **(C)** stomatal conductance, **(D)** water use efficiency, **(E)** EL in leaves, **(F)** EL in roots, **(G)** H_2_O_2_ in leaves, **(H)** H_2_O_2_ in roots, **(I)** MDA in leaves, and **(J)** MDA in roots of two barley genotypes Annora (salt sensitive) and Awaran 02 (salt tolerant). Values are expressed as means of three replicates with standard deviations. Different letters indicate that the values are significantly different at a *p*-value < 0.05.

#### Effects of zinc nanoparticles on oxidative stress parameters

The results revealed that the EL, H_2_O_2_, and MDA contents in barley shoots and roots were enhanced with increasing concentration of salinity (Figure 3), and maximum oxidative injury by salinity stress was observed in the sensitive barley cultivar (Annora) as compared with the tolerant cultivar (Awaran 02). On the other hand, applying ZnO NPs significantly reduced oxidative stress in both barley cultivars. The maximum reduction in oxidative stress was observed with the foliar application of ZnO NPs compared to the soil application of ZnO NPs (Figure 3).

#### Effects of zinc nanoparticles on antioxidant enzyme activities

The impact of ZnO NPs on antioxidant enzyme activities (SOD, POD, CAT, and APX) in barley leaves and roots under salinity stress is presented in Figure 4. The activities of all aforementioned antioxidant enzymes significantly reduced under salinity stress, and the lowest contents were observed in the sensitive genotype (Annora) in comparison with the tolerant genotype under salinity stress. However, the application of ZnO NPs significantly improved the antioxidant enzyme activities, and a maximum increase in the antioxidant enzyme activities was observed by the foliar application of ZnO NPs as compared to the soil application of ZnO NPs (Figure 4).

The article "Mitigation of salinity stress in barley genotypes with variable salt tolerance by application of zinc oxide nanoparticles" was retracted in 2024. Reasons: compromised peer review; unreliable results or conclusions.

**FIGURE 4:** Effects of different concentrations of NaCl (0 and 100 mM) and ZnO NPs (0, 100 mg kg^–1^ soil, and 100 mg L^–1^ foliar) on **(A)** SOD in leaves, **(B)** SOD in roots, **(C)** POD in leaves, **(D)** POD in roots, **(E)** CAT in leaves, **(F)** CAT in roots, **(G)** APX in leaves, **(H)** APX in roots of two barley genotypes Annora (salt sensitive), and Awaran 02 (salt tolerant). Values are expressed as means of three replicates with standard deviations. Different letters indicate that values are significantly different at a *p*-value < 0.05.

## Discussion

Various researchers reported that salt stress dramatically reduces plant growth, number of leaves/plant, root length, and plant biomass by disturbing the ion balance and osmoregulation in plants (Sharmin et al., 2021; Zhu et al., 2022). In this study, salinity stress (100 mM) decreased the shoot length, root length, number of leaves per plant, leaf area, and shoot and root dry biomass in barley cultivars (Supplementary Table 1). When soil salinity reaches a certain threshold, root growth is inhibited, resulting in a decrease in WUE, water uptake capability, leaf water potential, and transpiration rate under salt stress (Mushtaq et al., 2020; Ibrahimova et al., 2021; Kamran et al., 2021). Application of 100 mM NaCl drastically reduced the net photosynthesis rate and chlorophyll concentration in barley leaves (Supplementary Table 2; Table1). Stressed plants close their stomata to conserve water in the leaves, resulting in less CO_2_ entry and a slower rate of photosynthesis, which reduce the amount of photosynthetic products generated directly or indirectly (Bharath et al., 2021). Salt stress reduces turgor strain, resulting in a significant reduction in cell growth, cell elongation, cell division, and, as a result, overall plant growth (García-Caparrós and Lao, 2018; Rizwan et al., 2018; Mushtaq et al., 2020).

Results showed that plants treated with ZnO NPs recovered the plant growth under salinity stress as compared to its respective control. Zinc fertilization improves a plant ability to withstand salt, and ZnO NPs can help plants cope with the negative effects of abiotic stress due to the high concentration of sodium in soil (Sturikova et al., 2018). This beneficial effect of foliar application may be due to important role of Zn in plant biological and metabolic activities, such as stimulating enzymes, cell elongation and enlargement, nitrogen metabolism, photosynthetic pigments, preserving the structural integrity of plant cell membranes, and phospholipid accumulation (Rizwan et al., 2019; Adrees et al., 2021; Czyżowska and Barbasz, 2022). Exogenous application of ZnO NPs may reduce the leaf and root EL, further enhancing the antioxidant enzyme activities than treatments without ZnO nanoparticles. The increased production of antioxidant enzymes and reduced EL with ZnO NPs may enhance the barley growth treated with a high sodium concentration. The effectiveness of ZnO NPs is also determined by their ability to penetrate the plant cell through the natural Nano pore (stomata) in the leaves, which may enhance metabolic activities and, as a result, plant development (Rossi et al., 2019). The exogenous application of ZnO NPs improved the shoot length, root length, number of leaves, leaf area, shoot dry weight, and root dry weight even at 100 mM sodium concentration in both cultivars (Figure 1). The ZnO NPs reduced sodium toxicity in the plants, restored chlorophyll contents, and improved photosynthesis. Adding ZnO NPs to plants increased photosynthetic activity, improved carbohydrate and by-product metabolism, and increased plant tolerance to salt stress. ZnO NPs application reduced the sodium concentrations in plants than respective treatments without nanoparticles. Furthermore, Zn increases the biosynthesis of the growth regulator IAA, which promotes cell division, cell elongation, and mineral absorption, resulting in increased plant growth (Fernández and Brown, 2013; Zhang et al., 2021).

The article "Mitigation of salinity stress in barley genotypes with variable salt tolerance by application of zinc oxide nanoparticles" was retracted in 2024. Reasons: compromised peer review; unreliable results or conclusions.

Nanoparticles have a greater capacity and dynamic to be absorbed, translocated, assimilated, and accumulated in plants than their bulk counterparts due to their smaller size. Nanoparticles can pass through the cell wall and plasma membrane, and their high specific surface area and higher uptake rate explain why they are more efficient than bulk types in the application (Mehrabani et al., 2018; Lang et al., 2021). The gradual release of Zn ion from the nanoparticles, which supplies a long-term provenance of Zn and helps escape toxicity by sudden uptake of Zn by plants at high concentrations, may be responsible for the various physiological effects of the foliar supply of ZnO NPs (Wang et al., 2018). The increase in plant growth with nanoparticle application may be attributable to increased nutrient production, reduced soil toxicity induced by overuse of fertilizers, and increased antioxidant enzyme activity, which helps protect plants from injury caused by free radicals (Rajput et al., 2021). The present findings revealed that salinity enhanced ROS production while reducing the antioxidant enzyme activities (Figures 3, 4). Salinity stress results in ROS production; damage of nucleic acids, lipids, and proteins; and, ultimately, cell death. Cell damage might be due to ROS-induced lipid peroxidation of unsaturated fatty acids and impaired membrane functions (Demidchik et al., 2014; Zeeshan et al., 2020; Etesami et al., 2021). Furthermore, Kumar et al. (2017) also reported that salinity stress increased the contents of H_2_O_2_, EL, and MDA. This overproduction of ROS might have weakened the defense of barley plants by overcoming the activities of antioxidant enzymes such as SOD, POD, CAT, and APX activities, as evident by the present study. However, the exogenous application of ZnO NPs alleviated oxidative stress induced by salinity stress by improving plant defense and by enhancing the antioxidant enzyme activities. The present results are also supported by Hussein and Abou-Baker (2018), in which nano-zinc alleviated salinity stress in cotton plants. Moreover, salinity stress has been reduced by the application of ZnO NPs in different plants such as in *Brassica napus* (El-Badri et al., 2021), mango trees (Elsheery et al., 2020), lupine (Abdel Latef et al., 2017), and tomato plants (Hosseinpour et al., 2020), which might be due to improvement in the antioxidant enzyme activities with the exogenous application of ZnO NPs. A detailed graphical presentation is given in Figure 5, which depicts the effects of exogenously applied ZnO NPs and salinity stress on the plant growth and physio-biochemical attributes of barley.

The article "Mitigation of salinity stress in barley genotypes with variable salt tolerance by application of zinc oxide nanoparticles" was retracted in 2024. Reasons: compromised peer review; unreliable results or conclusions.

**FIGURE 5:** Graphical representation of the effects of exogenously applied ZnO NPs and salinity stress on the plant growth and physio-biochemical attributes of barley.

## Conclusion

Based on the plant growth and morphology, Awaran 02 was found as the most resilient genotype, and Annora turned out to be most sensitive during initial screening, which suggest the variations in salinity sensitivity within a species. The application of ZnO NPs to sensitive (Annora) and tolerant (Awaran 02) barley genotypes under salt stress demonstrated the importance of nanoparticles in reducing salt stress in barley. Application of ZnO NPs reduced the uptake of Na^+^ ions and increased the uptake of Zn in salinity-affected plants, which ultimately increased plant growth, biomass, and photosynthesis activity. Application of ZnO NPs mitigated salinity stress in the barley plants by suppressing the production of ROS and stimulating the production of antioxidant enzymes. The findings confirmed that foliar application of ZnO NPs is more significant than soil application due to the direct absorption of zinc by leaves during foliar spray. The use of nanoparticles could be a promising approach to cultivate the crops on salinity-affected soil and strengthen the plans to withstand the salinity stress. However, very little information is available about the action mechanism of NPs with sodium ions, the permissible limit of NPs, and the ecotoxicity in edible crops. Further comprehensive studies are required for the field-scale application of ZnO NPs in saline soils.

The article "Mitigation of salinity stress in barley genotypes with variable salt tolerance by application of zinc oxide nanoparticles" was retracted in 2024. Reasons: compromised peer review; unreliable results or conclusions.

## Data availability statement

The original contributions presented in the study are included in the article/Supplementary material, further inquiries can be directed to the corresponding authors.

## Author contributions

BA and MZ-U-R: conceptualization. BA and MR: data curation. WI: germplasm acquisition. KQ, MJ, SS, MSh, and AH: formal analysis. KQ, MJ, and SS: funding acquisition. MSh and WI: investigation. BA and MSh: methodology. MHS and SA: resources. BA and SA: supervision. MR: validation. MHS, AH, and MZ-U-R: visualization. BA, MT, MSa, SA, AH, MR, WI, and MZ-U-R: writing–original draft. MHS, KQ, MJ, SS, SA, MSa, and MT: writing–review and editing. All authors have read and agreed to the published version of the manuscript.
